# Construction of Smart City Street Landscape Big Data-Driven Intelligent System Based on Industry 4.0

**DOI:** 10.1155/2021/1716396

**Published:** 2021-12-14

**Authors:** Zhe Li, YuKun He, XinYi Lu, HengYi Zhao, Zheng Zhou, YinYin Cao

**Affiliations:** ^1^School of Architecture, Southeast University, Jiangsu 210096, China; ^2^Graduate School of Engineering, Kyoto University, Kyoto 606-8501, Japan

## Abstract

With the application of engineering management in smart city construction under Industry 4.0, the intelligent design of urban street landscape has attracted extensive attention. Affected by the low intelligent level of traditional landscape design, the existing urban landscape composite system has difficulty in meeting the needs of smart city construction. Therefore, this paper proposes the construction of street landscape big data-driven intelligent decision support system based on Industry 4.0. Based on the complex network theory, this paper analyzes the structure, links, nodes, driving forces, and functional requirements of urban street landscape and then puts forward the construction content and implementation method of urban street landscape intelligent decision support system. The system consists of four aspects: intelligent infrastructure, service, protection and maintenance, and management and evaluation system. Its implementation not only reflects the cooperation and effective application of intelligent technology in each stage of street landscape construction, but also provides reference for the application of engineering management in other fields under Industry 4.0.

## 1. Introduction

Based on the connectivity provided by the Industrial Internet of Things (IIoT) and the use of a variety of digital technologies such as cloud computing, big data, and artificial intelligence, Industry 4.0 is proposed as a new stage of industrial maturity [1, 2]. These technologies have produced an industrial method of automation and interconnection involving objects, products, and people, thus achieving a higher level of industrial performance [3]. With the application of engineering management in smart city construction under Industry 4.0, the intelligent design of urban street landscape also rises and develops rapidly. Meanwhile, “intelligent” development has become the new trend in modern society due to the advancement of information technology represented by the Internet. The smart city emerges in this context, which can detect, analyze, and integrate the key information of urban core operating systems using information and communication technologies, thus making intelligent responses to various needs covering people's livelihood, environmental protection, public security, urban services, and industrial and commercial activities [4]. The intelligent urban management and operation relying on advanced information technologies can effectively solve the complex urban problems and promote the harmonious and sustainable urban development [5].

As an important part of smart city construction, landscape architecture is also facing opportunities and challenges brought by the intelligent process. Smart gardens changing the construction, operation, and management modes of traditional gardens can effectively improve the efficiency in landscape garden industry, realizing the normalization, standardization, digitization, networking, and intelligence of garden construction [6]. The typical scenario of urban street landscape has significant effects on shaping the urban image. By selecting street landscape as the entry point of smart gardens, this paper aims to explore the needs of urban street landscape and discuss the intelligent system construction and implementation means, in order to provide reference for the construction of urban street intelligent systems [7, 8]. However, under Industry 4.0, in the process of intelligent city construction, how to effectively use new technologies such as big data and Internet of Things, as well as the interconnection between urban street landscapes after 5G network integration, has attracted people's attention to the security and anti-network attack stability of these systems.

## 2. Related Works

In the construction of urban street landscape intelligent system, “urban street” refers to the urban road equipped with sidewalks, municipal utilities, and various buildings on both sides in the overall length or most sections. As one of the subsystems under the future urban open complex giant system, the nature, function, form and structure of urban street are more complex than traditional urban road. Urban street serving as the most basic public urban space focuses on the citizens' life and humanized experience, which facilitates the interpersonal communication and interactions via emotional sustenance as well as playing an irreplaceable role in shaping the urban charms and vitalizing the economic development [9, 10].

Relying on the complex network theory and “Internet +” thinking, the smart landscape cooperates with new-generation information technologies such as Internet of Things, big data cloud computing, mobile Internet, remote sensing, and information intelligent terminal, obtains time-domain advantages, and responds quickly to social and natural activities carried in the landscape space. Integrating the spatial domain of modern ecological landscape into the large database achieves the intelligent connection between scattered social activities and needs of human beings, nature and landscape space for the interactive perception, and cognition and communication and improves the utilization and sharing rate of various scattered landscape resources, thus promoting the intelligent construction, service, and management of landscapes [11, 12].

The design of intelligent street landscape systems shall be based on the comprehensive consideration of user needs, greening landscapes, and basic street functions, through the Internet of Things, web services, and virtualization technology. The basic attributes, characteristic parameters, status, and other information of various street landscape elements are dynamically and intelligently sensed and accessed in real time, to build street space intensively. Through processing the information perceived by the landscape intelligent system, data collection, integration, analysis, processing, and feedback are realized under the mapping of landscape resources in urban streets. On the premise of ensuring the basic functions of the road, people's travel safety, life, and social security should be guaranteed, which provides conditions for the scientific, rapid, comprehensive, and visual development of urban street landscape design and management.

The construction of intelligent systems for urban street landscape based on complex network theory and the integration of smart landscape concept into the traditional urban street landscape indicate further improvement, which shall meet the requirements for intensive intelligent spaces, multiple interactive experience, and green ecology of energy conservation [13, 14].

## 3. Composition of Intelligent Systems for Urban Street Landscape

In order to cope with the multiple landscape needs under the complex system of urban streets, the intelligent street landscape system based on the complex network realizes the intelligent supply-demand matching of street landscape space services from the three levels of landscape facilities Internet of Things, service Internet, and user Internet.

The construction of street landscape intelligent system mainly involves four aspects: intelligent infrastructure, intelligent service, intelligent protection and maintenance, and intelligent management and evaluation.

### 3.1. Intelligent Infrastructure

Intelligent infrastructure is the physical layer and the foundation of street landscape intelligent systems. The infrastructure of street landscape intelligent systems shall proactively provide the information and services desired in addition to the basic functions and be available to correlate with other facilities and even users for the formation of a complete intelligent network featuring information interaction and function linkage, thus completing the virtualization and service-oriented information interaction and functional linkage of the intelligent information system.

#### 3.1.1. Information Infrastructure

Information infrastructure is the basis of intelligent street landscape, covering the electric information screen shown in Figure 1, multimedia touch screen terminal shown in Figure 2, intelligent monitoring, intelligent broadcasting, help facilities, security facilities, and landscape performance facilities. The foundation of infrastructure construction lies in the sound network transmission and communication networks, and relevant facilities shall be arranged in the densely populated areas (e.g., road entrances, parking lots) to facilitate the service provision such as information inquiry and satisfy the important requirements of easy identification and convenient use. The service scope of facilities with special functions (e.g., help facilities and security facilities) shall cover the entire street area, as well as focusing on the locations along main/secondary trunk roads and various open spaces, activity sites, and surroundings of green landscapes [15].

#### 3.1.2. Data Infrastructure

Data cognition is the core of intelligent street landscape development. The data infrastructure is used to collect and integrate street landscape data, achieving the intelligent street landscape construction by providing the users and managers with comprehensive and intuitive information based on the integration and analysis of multisource data (basic/business/service databases).

Basic database clarifies the spatial location and surrounding environment of urban street landscape for the precise positioning of smart landscape. Business database has multiple subdatabases covering the special data, system planning and management, monitoring management, and industry management available for the precise and whole-process collection of street landscape data. Service database can provide the popular science knowledge about smart street landscape for the public and facilitate the review of various urban green spaces and scenic spots by potential travelers [16].

#### 3.1.3. Observation Points of Street Green Space Ecosystem

Based on the ecological requirements of the street landscape intelligent system construction, ecological observation of the street is an effective measure to achieve this goal. Using RFID (radio frequency identification) technology, the real-time update of spatial ecological information of street landscape can be realized, and the location of vegetation, structures, and buildings can be monitored online. Special sensors and wireless sensor networks for street landscape ecological observation can effectively realize real-time data acquisition and transmission. Real-time monitoring of the street green space ecosystem can help with maintenance and management of the green landscape. Furthermore, the obtained ecological econometric characteristic data can aid in the formation of quantitative analysis results of the street landscape space, resulting in better landscape and ecological effects from green space maintenance and management, Figure 3.

### 3.2. Intelligent Service

The service object of the intelligent street landscape systems is the streetscape users. The construction of intelligent service system is based on Internet functions, which can realize the dynamic matching of the user's needs. From the perspective of users, in the process of system construction, our goals and demand motivation can be evaluated, and the service content can be derived dynamically.

In terms of qualitative or quantitative data, managers could be provided with genuine feelings, opinions, and suggestions generated by the public in the service experience. With the help of dynamic characteristics analysis of smart infrastructure, a reliable method for demand forecast management is provided. Thus, public involvement can be achieved, and the quality of the service improves continuously [17].

#### 3.2.1. Network Service Platforms

Network service platforms are the basis for intelligent service and the guarantee for intelligent linkage with other service facilities. The construction of portals serving the public shall cover various services such as bus routes, e-maps, traffic notices, travel tips, and road service calls. In addition, the construction of mobile-based network service platforms (e.g., mobile apps, WeChat public accounts) shall also be emphasized to ensure the real-time content update and provide mobile users with street information services based on the shared portal resources.

#### 3.2.2. Basic Street Services

Basic street services are mainly the traffic, lighting, and other necessary basic services. For instance, the smart parking management system achieves the real-time monitoring of parking spaces and the intelligent guidance about available parking spaces based on the information inquiry of parking lots and spaces through various intelligent terminals such as smart phones. The construction of public transportation system shall ensure the timely release of bus information and certain functions (e.g., multimedia information release, passenger complaint) in combination with the special bus signal system for important bus corridors and the intelligent bus stations. The streets with heavy traffic flows shall be equipped with smart toilets, which are available for the information inquiry of location and real-time usage through various intelligent terminals (e.g., smart phones, multimedia touch screens). In addition, the intelligent lighting system subject to the independent sensing, timing, voice control, or remote control of intelligent terminals shall also be arranged for the smart control of landscape lighting in different areas [18], Figure 4.

#### 3.2.3. Road Navigation

The intelligent terminals (e.g., smart phones, multimedia touch screens) and multilanguage terminals for self-service navigation shall be arranged to facilitate the inquiry of street and surrounding-area e-maps and tour route planning as well as the scenic spot/plant introduction using QR code/RFID technologies [19].

#### 3.2.4. Information Release

An interactive information system shall be established to provide life, service, business, and medical information for citizens, with various network service platforms serving as the channels for street information release, covering the street information, real-time road conditions, toilet usage, spare parking spaces, restaurant usage, and other basic information; climatic information (e.g., street temperature, humidity) and health information such as negative oxygen ion content in key areas Figures 5, flowering phase, and news and cultural event notices (e.g., lectures, exhibitions, festival activities, fitness events) at sites along the street; and information of emergency responses.

#### 3.2.5. Personalized Services

Personalized services available at various network service platforms can meet the street use demands of different people [20], for instance, the online adoption of plants along the street, and regular pushing of plant growth status and daily conservation information; pushing of intelligent infrastructure, location awareness, environmental monitoring index analysis, online security, and health information via the Internet; and application of intelligent technologies based on the users' different needs of travel and fitness.

#### 3.2.6. Consulting/Complaint Services

Compared with the traditional consulting/complaint services, the services provided through the intelligent system are more convenient and efficient, and multiple channels (e.g., street intelligent terminals, consulting/complaint pages, mobile terminals) are available for the public. The intelligent system of linkage service can achieve the unified receipt and instant feedback/response to consultations and complaints from telephones and network terminals.

#### 3.2.7. Virtual Experience

In order to improve the user experience, a multimedia experience center focusing on historical districts shall be constructed using multiple technologies (e.g., GIS, VR, and multimedia) for the display of historic landscapes, original natural features, and historical changes. The 3D panorama/reality enhancement display technology and 360°/720° real-life photos or videos can be utilized to create the virtual blocks for digital virtual tours that are available at portals and terminal devices (e.g., multimedia touch screens, smart phones) [16, 21].

### 3.3. Intelligent Protection and Maintenance

Intelligent protection and maintenance are the function expansion of the user Internet based on the Internet of Things of landscape facilities. Dynamically generate landscape maintenance needs based on smart infrastructure, and dynamically match landscape maintenance needs with landscape maintenance services through the Internet of Things technology. Realize the informatization and intelligence of the protection and maintenance process, provide visual guidance on daily maintenance process and key technology, and the responsible personnel and stages could be specified for the real-time recording of maintenance process and information [22].

#### 3.3.1. Green Space Protection and Maintenance

Green space protection and maintenance are the key to intelligent protection and maintenance, covering the digital recording, monitoring, and control of boundaries and green resources including the main plants and facilities. The important spots and key facilities shall be equipped with 3D scenes for inspection and comparison via intelligent terminals, mainly involving the plant irrigation and fertilization, pest and disease and freezing damage management, and intelligent cultivation.

Environmental monitoring and intelligent irrigation system can provide effective services for intelligent plant irrigation and fertilization management. The digital data processing of soil nutrients can maximize the effects of water-saving and precise irrigation, scientific management, and low-carbon maintenance [23, 24]. The construction of soil monitoring subsystem is available for the real-time monitoring of ambient temperature and humidity, wind direction, rainfall, and illuminance in the surrounding environment Figure 6, with the sensing facilities adopted for real-time detection of soil moisture, fertility, and other green space indexes. Maintenance decision-making depends on the IoT-based intelligent analysis and sorting of monitoring data received by servers [25]. In addition, the sprinkling and dropper systems are used for the automatic irrigation and fertilization and other intelligent applications, and the landscaping personnel can also search and receive monitoring data and warning information via computers and mobile phones Figure 7.

The GPS positioning and FRID technologies shall be adopted for the control of plant diseases and pests, with the dynamic tracking system established to ensure the dynamic protection and monitoring of green plants as well as help technicians locate the areas of pests and diseases at first time. The implementation of “prevention-first” principle by each institution responsible for plant management and protection targeting the necessary early warning of pests and diseases within all periods can greatly reduce the prevention costs and probability of large-scale pests and diseases [26]. Early warnings for the freezing damage management shall be issued in advance based on the weather conditions, providing the scientific basis and guidance for plant winter protection.

The intelligent technology-based seedling planting and cultivation shall make full use of the IoT and spatial information integration technologies. The partitional measuring of regional soil quality, hydrological conditions, and microclimate factors at the stage of planting planning provides the definite data basis for breeding and rapid formulation of cultivation schemes. At the same time, a tree full cycle database shall be established for plant tracking and data sorting in the whole process, as well as the records of seedling archives, tree transplantation, and maintenance information. Intelligent cultivation can effectively prevent the challenges faced by the traditional seedling cultivation (e.g., improper layout of trees, unsatisfactory production or waste of seedlings).

#### 3.3.2. Heritage Protection and Maintenance

Both natural heritage and cultural heritage involve heritage protection and maintenance, including ancient and famous trees and cultural relics. For the ancient and famous trees, the high-definition photos shall be obtained based on the precise coordinate positioning via monitoring and RFID technology in addition to the normal maintenance measures, and mastering relevant detailed information will facilitate the data calling, plant protection, document management, maintenance, and rejuvenation monitoring. Digital modeling based on the growth environment of ancient and famous trees also facilitates the accurate analysis of protection measures Figure 8. For the cultural relics and historical sites surrounding the street, the 3D data model shall be constructed to enhance the protection. The ancient buildings shall be equipped with stress-strain sensors for deformation monitoring and risk assessment [27].

### 3.4. Intelligent Management and Evaluation System

Scientific and comprehensive management measures are an important prerequisite for realizing the sustainable development of streetscapes. Quantitative evaluation mechanism is an effective objective to judge the effectiveness of streetscapes.

How to effectively integrate various scattered landscape management resources and coordinate various quantitative evaluation parameters to achieve the best match between street landscape management and demand is the key problem. Hence, quantitative data-driven evaluation and control system is ultimately conducive to the continuous optimization of landscape effects.

#### 3.4.1. Intelligent Management

The comprehensive and scientific management shall take account of internal office work, gardening business, street security, and other related factors.

Office automation (OA) system can improve the overall efficiency of internal office work, covering process management, e-mail, document management, document circulation, approval management, working calendar, notice announcement, personal information maintenance, conference management, and attendance management.

In terms of the gardening business management, video monitoring, RFID, and infrared sensing technologies shall be adopted for the real-time perception of changes in street green resources, infrastructure, and traffic flows, as well as the automatic collection, adjustment, and update of street landscape data. The real-time monitoring of street landscape can achieve precise management and prevention against vandalism and damage caused by natural disasters.

Street security cannot be neglected considering the special traffic function of urban street with public spaces. The construction of integrated street control platform makes the daily operation monitoring and emergency command and dispatching possible, providing basic support for navigation and guidance based on the location services of GIS and satellite positioning systems [28]. Nowadays, the rapid development of information technology also facilitates the dynamic monitoring of public opinions released via key media, forums, blogs, and Weibo platform; extraction of relevant information; and timely warning/treatment of potential crisis events in accordance with predetermined strategies.

#### 3.4.2. Intelligent Evaluation System

The evaluation of self-diagnosis by intelligent evaluation system aims to provide reference for further development. Moreover, reasonable performance evaluation can not only measure the achievements of street landscape construction and find out the existing problems, but also provide important guidance for the continuous improvement of street landscape intelligent system.

Establishment of the complete, scientific, and effective evaluation system shall be based on the existing urban gardening standards, with the relevant street smart landscape indicators integrated into the system by means of spatial layers, forms/tables, document uploading, and image attachments for real-time computing and result judgment/analysis [29], Table 1.

## 4. Technical Means of Intelligent Systems for Urban Street Landscape

Intelligent technology refers to a specific technology or method used in the construction of an intelligent urban streetscape system. Internet of Things, spatial information integration, virtual reality and visualization technology, digital technology, etc. can solve the following problems in the construction of streetscape system under the condition of urban complex giant system:

1. How to manage, digitize, and integrate information from scattered roads efficiently and precisely, in order to realize the effective distribution and dynamic overall grasp of the streetscape service capabilities.
2. How to coordinate the relationship between the geographic space, data flow, time distribution, hardware network, and user needs of the streetscape intelligent system, in order to realize the spatial mapping between complex streetscape resources and intelligent system service capabilities [30].

Emergence of the most representative IoT technology in the intelligent process has led the transformation of information age into an intelligent era. The all-inclusive IoT technology involving radio frequency identification (RFID), infrared sensor, and sensor-laser scanner solves numerous urban problems via interconnection of things after the Internet-based information connection [31].

Spatial information reflects the spatial distribution characteristics of geographic entities, and the spatial information integration technology involving remote sensing (RS), geographic information system (GIS), and global positioning system (GPS) can reflect the topographical features of all sites more concretely and objectively at the macro level and achieve precise quantification and data digitization for in-depth research and analysis [32].

VR technology integrates multiple techniques features in good experience of immersion, interaction, and conception, covering the real-time 3D computer graphics, 3D wide-angle (wide-field) display, tracking of the viewer's head/eyes/hands, tactile/force feedback, stereo effects, network transmission, and voice input/output [33].

The basic process of digitization involves the transformation of all complex and changeable information into measurable data, digital data modeling for binary code conversion, and input into the computer for unified processing [34]. At present, the digital technology is widely used in various industries, and the digitization serving as the predecessor of intelligent technologies shall be utilized continuously in the intelligent era.

## 5. Prospects of the Construction and Application of Intelligent Systems for Urban Street Landscape

To achieve the successful construction of street landscape intelligent systems, the mutual mapping of complex system and complex network of street landscape needs to be realized. Therefore, the above intelligent means must be implemented combined with the actual stages of street landscape construction in practice.

### 5.1. Planning and Design Stage

The early stage of planning and design provides direct guidance for the mid-term construction and post-management of landscape construction. The application of intelligent means such as the Internet of Things, virtual reality, and visualization technology at the planning and design stage can realize more scientific and rational street landscape design.

In terms of on-site investigation, the traditional investigation methods have large workload and large error, and most of them are completed on the basis of on-site inspection and surveying and mapping, combined with the existing data. In addition, the traditional street design focusing on-site plane lacks the 3D-space and humanized thinking in terms of vertical design, construction scale, and detailed design. On the contrary, the intelligent landscape construction can realize the targeted integration of IoT and spatial information technologies into the site survey, with the precise positioning of street location and surrounding land uses utilizing the IoT sensing nodes [35]; moreover, the spatial information technology enables the designer to understand the connections between overall street appearance/style and urban image more comprehensively and accurately Figure 9.

### 5.2. Construction Stage

The construction quality directly affects the smooth implementation of the preliminary design and the cost of later maintenance and management. Due to the problems of inaccurate calculation of quantities, unconstrained construction, and limited professional quality of most construction personnel in traditional garden construction, there are often some deficiencies in construction quality compared with the expected effect.

The intelligent street landscape construction can ensure the rational resource allocation and construction efficiency through the in-depth survey of on-site environmental factors (e.g., soil quality, hydrological conditions, wind force, atmospheric pressure) using the sensing and RFID systems of IoT technology and the corresponding construction schemes and regulations. The application of spatial information integration technology and sensing system makes precise and rapid data positioning based on construction drawings possible at the stage of fixed point setting-out. The multispace model using VR technology enables the construction personnel to understand the design intention in an intuitive manner during construction, thus ensuring the realization of design effects. The application of IoT sensing system upon project acceptance for data measurement and quantitative analysis of engineering effects, combined with the direct data transmission to the auditor's mobile devices using mobile Internet technology, guarantee the strict project acceptance [36], Figure 10.

### 5.3. Green Plant Cultivation and Conservation Stage

Conservation management can maintain and guarantee the landscape effects after gardening construction. The traditional plant cultivation and conservation have certain shortcomings, e.g., unsatisfactory professional quality of management personnel and conservation measures of low technical contents.

The intelligent plant cultivation and conservation integrating IoT technology ensure the effective improvement of conservation efficiency and effects with reduced cost. In order to make proper use of local conditions, the sensors shall be used to measure environmental factors (e.g., humidity and soil quality) at the cultivation stage, and the original manual sprinkling shall be replaced by the sprinkling/drip irrigation system with time-frequency sensors to detect the soil moisture and facilitate the intelligent control [37]. In terms of fertilization, winter protection, and wind protection, the digital model established based on the plant growth environment can realize the precise analysis of proper measures in different periods to ensure the normal plant growth and optimal effects Figure 11.

## 6. Conclusion

Applying intelligent means in urban street landscape design and integrating street landscape intelligent system into smart city construction can actively promote urban development. Procedures starting from scheme design and project construction to maintenance management, technology introduction, and formulation of comprehensive and effective strategies are the key to the successful construction of street landscape intelligent system based on complex network. In addition, the construction of street landscape intelligent system also provides a platform for public participation and governance. The public can easily and quickly obtain information through such intelligent systems and use improved consultation/complaint services to give timely feedback to managers, which indicates that public participation has been significantly improved [7, 38, 39]. In short, the street landscape intelligent system based on complex network theory provides an advanced and sustainable construction mode for the future urban complex street system. In the context of Industry 4.0, with the rapid development of big data and the Internet of Things, more in-depth research in the future should aim to integrate the street landscape intelligent system into the construction of smart city and build a perfect street landscape intelligent system.

## Figures and Tables

**Figure 1:** Electronic information screen.

**Figure 2:** Multimedia touch screen terminal.

**Figure 3:** Ecosystem observation facility.

**Figure 4:** Basic street services.

**Figure 5:** Street climatic information and health information.

**Figure 6:** Soil monitoring subsystem.

**Figure 7:** Intelligent irrigation system.

**Figure 8:** Digital monitoring of ancient and famous trees.

**Figure 9:** Application of intelligent technologies at the planning and design stage.

**Figure 10:** Application of intelligent technologies at the construction stage.

**Figure 11:** Application of intelligent technologies at the green plant cultivation and conservation stage.

**Table 1:** Intelligent evaluation index.

Target layer	Control layer			
	Evaluation object	Weights	Indicator layer	Weights
Evaluation of intelligent urban street landscape (A)	Material element (B1)	0.38	Functional facilities (C1)	0.35
			Recreation facilities (C2)	0.3
			Plant landscape (C3)	0.15
			Paved landscape (C4)	0.2
	Open space (B2)	0.28	Spatial scale fitness (C5)	0.3
			Environment comfort (C6)	0.25
			Landscape interface suitability (C7)	0.23
			Activity type richness (C8)	0.12
			Activity time richness (C9)	0.1
	Environmental ecology (B3)	0.34	Landscape sensitivity (C10)	0.35
			Landscape suitability (C11)	0.33
			Landscape health (C12)	0.32

## Data Availability

The labeled datasets used to support the findings of this study are available from the corresponding author upon request.
